The article "Mechanical Properties of Blood-Mixed Polymethylmetacrylate in Percutaneous Vertebroplasty" was retracted in 2010. Reason: duplicate publication.

# Mechanical Properties of Blood-Mixed Polymethylmetacrylate in Percutaneous Vertebroplasty

**DOI:** 10.4184/asj.2009.3.2.45

**Published:** 2009-12-31

**Authors:** Dong Ki Ahn, Song Lee, Dea Jung Choi, Soon Yeol Park, Dae Gon Woo, Chi Hoon Kim, Han Sung Kim

**Affiliations:** * Department of Orthopedic Surgery, Seoul Sacred Heart General Hospital, Seoul, Korea.; † Biomedical Engineering Department, Yonsei University, Wonju, Korea.

**Keywords:** Filler, Bone cement, Vertebroplasty, Osteoporotic verterbral compression fracture

## Abstract

**Study Design:**

Mechanical study of polymethylmetacrylate (PMMA) mixed with blood as a filler.

**Purpose:**

An attempt was made to modify the properties of PMMA to make it more suitable for percutaneous vertebroplasty (PVP).

**Overview of Literature:**

The expected mechanical changes by adding a filler into PMMA included decreasing the Young's modulus, polymerization temperature and setting time. These changes in PMMA were considered to be more suitable and adaptable conditions in PVP for an osteoporotic vertebral compression fracture.

**Methods:**

Porous PMMA were produced by mixing 2 ml (B2), 4 ml (B4) and 6 ml (B6) of blood as a filler with 20 g of regular PMMA. The mechanical properties were examined and compared with regular PMMA(R) in view of the Young's modulus, polymerization temperature, setting time and optimal passing-time within an injectable viscosity (20-50 N-needed) through a 2.8 mm-diameter cement-filler tube. The porosity was examined using microcomputed tomography.

**Results:**

The Young's modulus decreased from 919.5 MPa (R) to 701.0 MPa (B2), 693.5 Mpa (B4), and 545.6 MPa (B6). The polymerization temperature decreased from 74.2℃ (R) to 59.8℃ (B2), 54.2℃ (B4) and 47.5℃ (B6). The setting time decreased from 1,065 seconds (R) to 624 seconds (B2), 678 seconds (B4), and 606 seconds (B6), and the optimal passing-time decreased from 75.6 seconds (R) to 46.6 seconds (B2), 65.0 seconds (B4), and 79.0 seconds (B6). The porosity increased from 4.2% (R) to 27.6% (B2), 27.5% (B4) and 29.5% (B6). A homogenous microstructure with very fine pores was observed in all blood-mixed PMMAs.

**Conclusions:**

Blood is an excellent filler for PMMA. Group B6 showed more suitable mechanical properties, including a lower elastic modulus due to the higher porosity, less heating and retarded optimal passing-time by the serum barrier, which reduced the level of friction between PMMA and a cement-filler tube.

## Introduction

Vertebroplasty is a popular treatment for osteoporotic vertebral compression fractures, and various preventive strategies have been introduced to reduce the number and severity of complications. Bone cement leakage and embolism can occur when a lower viscosity cement is infused through a cement filling tube with a relatively small diameter^1^,^2^. The cement that leaks into the spinal canal or neural canal can cause stenosis, and a high polymerization temperature can cause severe thermal injury to the nerve tissue^3^,^4^. In addition, the vertebral body strengthened with the cement itself might induce an adjacent vertebral compression fracture^5^-^7^. To reduce these complications from vertebroplasty, there have been several reports on the ideal mechanical properties of the cement for vertebroplasty, including methods for infusing the cement with high viscosity and the use of cement with less strength and a lower polymerization temperature^8^-^10^. The porosity generated by filler materials may allow the release of antibiotics loaded in cement more easily but their Young's modulus should be decreased. On the other hand, the cement must be beneficial in vertebroplasty and have other modified properties, including a reduced setting time due to the faster polymerization time and the lower polymerization temperature^10^-^12^. This study examined whether mixing blood into cement can make the mechanical properties more suitable to vertebroplasty to reduce the number of complications.

## Materials and Methods

### 1. Materials and mixing methods

Exolent Spine (Elmdown Ltd., London, UK) contained 20 g (20 ml) of polymer and 9.2 g (8 ml) of monomer per one pack. The specimens were mixed in a operating room with a room temperature of 18℃ and 21% humidity with the cement preserved at room temperature for more than 24 hours. Six specimens were made in each group including the regular cement group (R) and blood-mixed groups (B2, B4, B6), which contained separately 2 ml, 4 ml, and 6 ml of blood in a single pack of cement, respectively. One researcher gave blood, which had a hemoglobin and hematocrit level of 16.7 mg/dl and 34.8%, respectively. It was sampled immediately before being mixed with the cement and should be mixed within a short time (about 1 minute after sampling) prior to hematoma formation. Cement was mixed evenly at a 2 Hz speed for approximately 45 seconds and more 15 seconds after mixing the blood. The mixed cement was transferred into a 20 ml regular syringe and filled into a stainless mold with a 10 mm inner diameter and a 30 mm height to make one block for the Young's modulus, and into three filler tubes with a 2.8 mm inner diameter and 215 mm height to measure the optimal passing-time. The cement remaining in the syringe was transferred into a bowel to measure the polymerization temperature and setting time. The cement block was easily separated by light impact with a rod after 24 hours when the cement specimen had hardened completely. The height and diameter was manipulated accurately with sandpaper and inspected with Venier Calipers (Mitutoyo, Kawasaki, Japan) with 0.05 mm accuracy. The same procedures were repeated six times to make six samples and collect the data in each group.

### 2. Study methods

The Young's modulus was measured using an Instron Micro-test system (Instron, Norwood, MA, USA) under a compressive speed and load of 5 mm/minutes and 2 kN, respectively. The Young's modulus was defined as the slope of the stress-strain curve. The displacement by load was measured at 20 Hz and the data collected was analyzed using Bluehill 2 software (Instron). The polymerization temperature reached a maximum after mixing the polymer and monomer, and was measured using an Infrared Thermometer (AR852B; ARCO, Guangzhou, China) under the condition of 0.9 emissivity and within 10 mm from the specimen for the optimal optic-distance ratio. The setting time was defined as the interval time from a mixing-start point to a point reaching polymerization temperature^12^. The optimal passing time was defined as the possible interval time for the cement with an optimal viscosity to pass through a filler tube with a inner diameter of 2.8 mm using a 20-50 N hand pushing pressure. The cement viscosity that could be passed by less than 20 N hand pressure showed more running fluid character, and the cement viscosity that could be passed with 20-50 N showed sticky, tenacious and malleable properties. The hardened cement that required more than 60 N hand pressure could not be passed through the cement filler tube and fixed to the pusher within the tube. Considering these properties as cement hardened, the optimal passing-time was determined to be the interval showing a certain viscosity equal to the 20-50 N hand pressure. The pressure passing viscous fluid through a tube was determined to be the viscosity coefficient and diameter of the tube^8^. A larger diameter tube has been already used for higher viscosity cement in order to allow easy passing clinically. Therefore, this study used a tube with a 2.8 mm inner diameter and 215 mm length, which is generally used for kyphoplasty. A zig was required to connect the filler tube and a digital pressure gauge, FGP-5 (NIDEC-SHIMPO Corporation, Kyoto, Japan) tightly and avoid unnecessary resistant pressure evoked by a sagged axis. The minimal pressure required to pass the cement through the tube was measured (Fig. 1). The porosity of the cement specimens was measured using SkyScan 1076 Micro-CT System (Skyscan, Aartselaar, Begium). The data was analyzed using the SPSS 15.0 (SPSS Inc., Chicago, IL, USA). The Young's modulus, polymerization temperature, setting time, optimal passing-time and porosity were compared statistically using a one-way ANOVA test to test the null hypothesis, and a Tukey's-b test with a Post Hoc multiple comparison test was used to identify differences between the groups.

## Results

The Young's modulus of group R, B2, B4 and B6 was 919.5±148.2 MPa, 701.0±76.1 MPa, 693.5±104.1 MPa, and 545.6±93.1 MPa, respectively. The Young's moduli of the Blood-mixed polymethylmetacrylate (PMMA) groups were significantly lower than that of group R. The more blood-mixed PMMA showed a lower modulus but the difference between the groups was not significant according to the Post Hoc multiple comparison test (Table 1). The polymerization temperature of group R, B2, B4 and B6 was 74.2±2.6℃, 59.8±2.2℃, 54.2±1.6℃, and 47.5±1.0℃, respectively. The blood-mixed PMMA groups showed a significantly lower polymerization temperature than that of group R. In addition, the polymerization temperature and setting time decreased with increasing amount of blood.

The setting time of the group R, B2, B4 and B6 was 1065±15 seconds, 624±8 seconds, 678±3 seconds, and 606±8 seconds, respectively. The optimal passing-time of group R, B2, B4 and B6 was 75.6±2.6 seconds, 46.6±2.3 seconds, 65.0±6.1 seconds, and 79.0±4.2 seconds, respectively. The optimal passing-time increased with increasing amount of mixed blood but the setting time decreased. The optimal passing-time of B2 was almost the same as that of group R in the Post Hoc test.

The porosity of group R, B2, B4 and B6 in micro-CT was found to be 4.2±0.6%, 27.6±1.7%, 27.5±1.4% and 29.5±1.6%, respectively. The blood-mixed PMMA groups showed similar porosity regardless of the amount of mixed blood according to the Post Hoc test. Micro-CT revealed micropores distributed evenly in the blood-mixed PMMA groups (Fig. 2).

## Discussion

Vertebroplasty with PMMA for osteoporotic vertebral compression fracture is considered to be very successful in that stabilization of fractured osteoporotic vertebral body and dramatic pain relief. However, with the increasing use of the procedure, many complications have been reported. One of them was adjacent vertebral compression fractures, which might be caused by outward factors including stress transferred from a treated vertebra with PMMA, poor sagittal balance and compensation of the upper body shifting after pain relief, intradiscal cement leakage, cement configuration and an infused volume in the vertebral body as well as an inward resistant factor, i.e. bone density^6^,^7^,^13^-^17^. The strength of PMMA was eight to forty times higher than that of the osteoporotic vertebra. Therefore, harder PMMA in the verterbral body could cause more stress transfer to the surrounding cancellous bone, causing continuous refracturing of a treated body or into the adjacent vertebral endplate, resulting in an additional vertebral fracture^5^,^18^. Lower modulus PMMA or PMMA substitutes are recommended to reduce the newly increasing stress transfer after vertebroplasty^19^,^20^. The optimal modulus of PMMA for vertebroplasty cannot be determined due to the combined mechanical effects of the variety of causative factors on the adjacent vertebral fractures. However, considering the strength of PMMA only, a sufficient volume of PMMA supporting both the upper and lower endplates in the vertebral body was reported to increase the level of stress transfer by 670% and 200% using 3,000 MPa and 100 MPa PMMA, respectively^21^. Therefore, the use of commercially available PMMA with a modulus of 1,000 MPa for verterboplasty can cause approximately 200-400% stress transfer. In addition, the modulus of osteoporotic vertebral body was considered in stress resistance. The elastic modulus of the osteoporotic vertebral body was reported to be 34 MPa, 804 MPa, and 670 MPa in cancellous bone, cortical bone and endplate, respectively^22^, and the early recollapse rate was reported to be 16% in vertebroplasty with lower modulus substitutes, such as calcium phosphate cement^23^. The optimal modulus of PMMA was the modulus near the vertebral body to prevent a treated veterbral body from refracture and reduce the increase of stress transfer. The polymer to monomer ratio was changed to reduce the modulus of PMMA by 19.5% from 2,210 MPa to 1,780 MPa, but could not reach the clinical requirements^11^. Fifty percent mixing with a radiopaque material could decrease the modulus by 95.7%, from 2,800 MPa to 120 MPa, but the result was also ineffective clinically because PMMA with such a low modulus could not recover the strength of a treated vertebra to the preinjured level^24^. These results showed that 4 ml and 6 ml blood mixed PMMA showed a modulus of 701 MPa and 545.6 MPa, respectively, which is similar to the modulus of cortical and endplate in an osteoporotic vertebral body.

The moduli and porosities of the blood-mixed PMMAs were unaffected by the volume of blood. The lack on an increase in porosity with increasing blood volume was due to the previous mixing of the polymer and monomer for 45 seconds, which might already produce a certain level of polymerization, and the mixing methods with the hands in which there could be a limitation of flourishing porosity over a certain point. The early mixing of blood and PMMA might allow considerable porosity to the blood-mixed PMMA, but more porous PMMA was not required. Overplus blood, on the other hand, which did not be mixed with PMMA, was shifted to the surface of PMMA and produced a larger plasma barrier on the PMMA specimen.

Porosity caused by the mixing of a filler can reduce the modulus of PMMA. A filler which is available in verterbroplasty to endow porosity, should have high viscosity, easy resorption and release from PMMA, water solubility, biocompatibility and biodegradability^10^. Boger et al.^10^ reported that when a pack of PMMA was mixed with sodium hyaluronate at a 35% (13 ml) volume ratio, it resulted in a 56% porosity, a decrease in modulus and polymerization temperature from 1,837 MPa to 477 MPa and from 68℃ to 41℃, respectively, which could prevent thermal injury to the surrounding soft tissues. A very small amount of sodium hyaluronate is already used in a bone substitute product. However, such a large volume of sodium hyaluronate might cause an embolism in the blood. Hence, the safety cannot be guaranteed except for topical use in those regions from which sodium hyaluronate could not be resorbed directly into the blood^25^.

A filler and additive mixed with PMMA can reduce the polymerization temperature. A filler might produce pores in PMMA, which can allow the polymerization heat to dissipate quickly, and an additive may induce a new polymerization reaction with a lower heat of reaction. One of the theories of pain relief by verterbroplasty was the thermal necrosis of the peripheral endings of the nerve fibers in the vertebral body. However, calcium phosphate cement with no exothermic effect can show similar pain relief. On the other hand, a microscopic study showed that micronecrosis around PMMA after verterbroplasty was due to a resorption process rather than to a foreign body reaction caused by PMMA reaction heating or radiopaque barium^26^,^27^. The central temperature of PMMA in polymerization reached 49-112℃, and the duration in which the temperature exceeded 50℃ lasted for almost 8 minutes, which might be enough to injure the nerve tissue. If PMMA with the emission of significant reaction heat leaked into the spinal canal, heat transfer could be mostly intercepted by the continuous flow of the cerebrospinal fluid (CSF), but the mass effect could provoke stenosing neurologic symptoms. However, it would cause thermal injury to the nerve tissue if it leaked into the neural foramen and bordered on a root ganglion without the flow of CSF. Therefore, the reaction heat in the polymerization of PMMA should be lower^3^,^4^,^28^,^29^. In the case of blood-mixed PMMA, the polymerization temperature was as high as 47.5-54.2℃, which is not believed to be enough to prevent thermal injury but the temperature may be decreased easily to a safe level on surrounding tissues in a shorter time than that of regular PMMA.

According to the Hagen-Poiseuille law, the pressure required in passing liquid PMMA through a filler tube is dependent on the viscosity of the PMMA in direct proportion^8^.



The setting time decreased in the blood-mixed PMMA, which is similar to the same results of various filler-mixed PMMAs. A decrease in setting times means that the viscosity is elevated faster and PMMA hardens earlier. Viscous PMMA should be passed through a filler tube of a smaller diameter during verterbroplasty rather than kyphoplasty. If the viscosity is elevated over a certain level and an optimal passing-point is missed, sufficient volume of PMMA could not be infused into the verterbral body and become stuck in the tube. However, the optimal passing-time of blood-mixed PMMA was lengthened in proportion to the volume of blood regardless of the shortened setting time, because of the plasma barrier formed on the surface of the PMMA specimen, which worked effectively as a lubricant between the PMMA and the tube. The optimal passing-time of group B6 was similar to that of group R but the setting time of group B6 was reduced by 43% compared to group R. Hence, the viscosity of group B6 was much higher than that of group R at the same point of infusion, which can clinically reduce the risk of extravasation from a vertebral body or an embolism of PMMA.

Micro-CT revealed micropores which were distributed evenly but not interconnected, so the PMMA and cancellous bone could not be suspected to be conglutinated in the processing of bone union.

In some point of view, bone substitutes were suspected to be replaced for PMMA even in treatment for osteoporotic vertebral compression fractures. Bone substitutes undergo a process of crystallization without an exothermic effect in the body temperature rather than polymerization. In addition, they can be resorbed by osteoclasts followed by the remodeling of host bone, and do not release toxic substances like the monomer in PMMA^20^,^30^,^31^. However, calcium carbonate cement was resorbed very early within two to four months after infusion, making unable to support a collapsed body for sufficient time^32^, and calcium phosphate cement has a risk of recollapse of the fractured vertebral body due to the very low strength^23^,^33^. Calcium sulphate cement can restore the treated vertebral strength to a similar strength through regular PMMA but it has also a risk of refracture of the treated verterbra due to the rapid resorption^34^,^35^. It is believed that the advantage of resorption and replacement of calcium phosphate cement by the normal host bone does not exactly mean the recovery of bone density and strength to those of the young and healthy vertebra that would be sufficient to prevent refracture of an osteoporotic vertebral body. In addition, the use of these substitutes carries a risk of embolism, and the disintegration tendency can deteriorate the pulmonary and arterial oxygen tension in the aqueous environment of continuous blood flow in a vertebral body in an experimental study^36^. Hydroxyapatite is believed to overcome the disadvantages of regular PMMA and calcium phosphate cement. However, its high viscosity can make handling and infusion more difficult and the resorption property can be obscure. Its use is not yet prevalent because of its cost effectiveness^37^,^38^.

There were several limitations in this study due to the aims of the study, which was focused on identifying the clinical problems and solutions during performing vertebroplasty, and the measurement criteria and methods were thought to be possibly affected by the subjective opinion by researchers. The optic-distance ratio must be considered when using an infrared thermometer as a noncontact measurement. The recorded temperature would have been lower than the real temperature if the temperature was measured far from the acceptable distance according to optic-distance ratio when the larger measured area was detected by a non-contact measurement method. An infrared thermometer calculates the average temperature over a certain area. The emissivity of PMMA was believed to be 0.8-0.9, which is similar to plaster or brick. Steinless showed lower emissivity. Therefore, the measured temperature would have been much lower than the real polymerization temperature if the polymerization temperature was measured on the surface of a steinless mold containing PMMA. Accordingly, more studies using similar instruments and objective methods would be done to overcome these limitations and more advisable and objective methods could be commented.

## Conclusions

Blood was used as a biocompatible filler to modify the properties of bone cement to make it more suitable to vertebroplasty by reducing the Young's modulus to that of the osteoporotic vertebral body and lowering the polymerization temperature. The blood-mixed cement is believed to have clinical benefits in vertebroplasty, in that a lower modulus can reduce the level of stress to the adjacent vertebrae. In addition, the lubricant effect of the plasma membrane can allow a high viscosity cement to pass smoothly under the same pressure for passing regular cement to reduce a risk of cement leakage and embolism. Furthermore, a lower polymerization temperature might also reduce a risk of thermal injury to the nerve tissue.

## Figures and Tables

**Fig. 1:** Methods for measuring the pressure-related manipulation time. A cement filler with a 2.8 mm diameter was connected to FGP-5. A jig can hold a cement filler tightly along the parallel axis to FGP-5 to prevent unexpected resistant pressure during cement-pushing.

**Fig. 2:** Micro-configuration on micro-CT. Blood-mixed polymethylmetacrylate's (2B, 4B and 6B) showed homogenous structures with fine regular pores.

**Table 1:** Homogenous subsets by Tukey B test

## References

[1] Chen JK, Lee HM, Shih JT, Hung ST (2007). Combined extraforaminal and intradiscal cement leakage following percutaneous vertebroplasty. Spine (Phila Pa 1976).

[2] Lim SH, Kim H, Kim HK, Baek MJ (2008). Multiple cardiac perforations and pulmonary embolism caused by cement leakage after percutaneous vertebroplasty. Eur J Cardiothorac Surg.

[3] Teng MM, Cheng H, Ho DM, Chang CY (2006). Intraspinal leakage of bone cement after vertebroplasty: a report of 3 cases. AJNR Am J Neuroradiol.

[4] Ahn DK, Choi DJ, Lee S (2009). Spinal cord injury caused by bone cement after percutaneous vertebroplasty: one case of long-term follow-up and the result of delayed Removal. J Korean Orthop Assoc.

[5] Frankel BM, Monroe T, Wang C (2007). Percutaneous vertebral augmentation: an elevation in adjacent-level fracture risk in kyphoplasty as compared with vertebroplasty. Spine J.

[6] Rohlmann A, Zander T, Bergmann G (2006). Spinal loads after osteoporotic vertebral fractures treated by vertebroplasty or kyphoplasty. Eur Spine J.

[7] Rohlmann A, Zander T, Jony, Weber U, Bergmann G (2005). Effect of vertebral body stiffness before and after vertebroplasty on intradiscal pressure. Biomed Tech (Berl).

[8] Loeffel M, Ferguson SJ, Nolte LP, Kowal JH (2008). Vertebroplasty: experimental characterization of polymethylmethacrylate bone cement spreading as a function of viscosity, bone porosity, and flow rate. Spine (Phila Pa 1976).

[9] Belkoff SM, Sanders JC, Jasper LE (2002). The effect of the monomer-to-powder ratio on the material properties of acrylic bone cement. J Biomed Mater Res.

[10] Boger A, Bohner M, Heini P, Verrier S, Schneider E (2008). Properties of an injectable low modulus PMMA bone cement for osteoporotic bone. J Biomed Mater Res B Appl Biomater.

[11] McLaren AC, McLaren SG, McLemore R, Vernon BL (2007). Particle size of fillers affects permeability of polymethylmethacrylate. Clin Orthop Relat Res.

[12] Chiu FY, Lin CF (2009). Antibiotic-impregnated cement in revision total knee arthroplasty: a prospective cohort study of one hundred and eighty-three knees. J Bone Joint Surg Am.

[13] Berlemann U, Ferguson SJ, Nolte LP, Heini PF (2002). Adjacent vertebral failure after vertebroplasty: a biomechanical investigation. J Bone Joint Surg Br.

[14] Lin EP, Ekholm S, Hiwatashi A, Westesson PL (2004). Vertebroplasty: cement leakage into the disc increases the risk of new fracture of adjacent vertebral body. AJNR Am J Neuroradiol.

[15] Tanigawa N, Komemushi A, Kariya S (2007). Relationship between cement distribution pattern and new compression fracture after percutaneous vertebroplasty. AJR Am J Roentgenol.

[16] Harrop JS, Prpa B, Reinhardt MK, Lieberman I (2004). Primary and secondary osteoporosis' incidence of subsequent vertebral compression fractures after kyphoplasty. Spine (Phila Pa 1976).

[17] Ahn DK, Lee S, Choi DJ (2009). The efficacy of kyphoplasty on osteoporotic vertebral compression fracture: a 1-year follow-up study. J Korean Soc Spine Surg.

[18] Lin WC, Lee YC, Lee CH (2008). Refractures in cemented vertebrae after percutaneous vertebroplasty: a retrospective analysis. Eur Spine J.

[19] Hu X, Zhai X, Hirt T (2009). A new concept for more biocompliant bone cements for vertebroplasty and kyphoplasty. Macromol Biosci.

[20] Grafe IA, Baier M, Noldge G (2008). Calcium-phosphate and polymethylmethacrylate cement in long-term outcome after kyphoplasty of painful osteoporotic vertebral fractures. Spine (Phila Pa 1976).

[21] Chevalier Y, Pahr D, Charlebois M (2008). Cement distribution, volume, and compliance in vertebroplasty: some answers from an anatomy-based nonlinear finite element study. Spine (Phila Pa 1976).

[22] Polikeit A, Nolte LP, Ferguson SJ (2003). The effect of cement augmentation on the load transfer in an osteoporotic functional spinal unit: finite-element analysis. Spine (Phila Pa 1976).

[23] Kim EH, Shin DH, Nho JW, Ryu KH (2007). Kyphoplasty with calcium phosphate cement (Calcibon(R)) in osteoporotic vertebral fracture. J Korean Soc Spine Surg.

[24] Boger A, Bisig A, Bohner M, Heini P, Schneider E (2008). Variation of the mechanical properties of PMMA to suit osteoporotic cancellous bone. J Biomater Sci Polym Ed.

[25] Hexig B, Nakaoka R, Tsuchiya T (2008). Safety evaluation of surgical materials by cytotoxicity testing. J Artif Organs.

[26] Togawa D, Kovacic JJ, Bauer TW (2006). Radiographic and histologic findings of vertebral augmentation using polymethylmethacrylate in the primate spine: percutaneous vertebroplasty versus kyphoplasty. Spine (Phila Pa 1976).

[27] Togawa D, Bauer TW, Lieberman IH, Takikawa S (2003). Histologic evaluation of human vertebral bodies after vertebral augmentation with polymethyl methacrylate. Spine (Phila Pa 1976).

[28] Belkoff SM, Molloy S (2003). Temperature measurement during polymerization of polymethylmethacrylate cement used for vertebroplasty. Spine (Phila Pa 1976).

[29] Kim KT, Suk KS, Kim JM, Park KC (2001). Root injury after percutaneous vertebroplasty in compression fracture: case report. J Korean Soc Spine Surg.

[30] Libicher M, Hillmeier J, Liegibel U (2006). Osseous integration of calcium phosphate in osteoporotic vertebral fractures after kyphoplasty: initial results from a clinical and experimental pilot study. Osteoporos Int.

[31] Sturup J, Nimb L, Kramhoft M, Jensen JS (1994). Effects of polymerization heat and monomers from acrylic cement on canine bone. Acta Orthop Scand.

[32] Cunin G, Boissonnet H, Petite H, Blanchat C, Guillemin G (2000). Experimental vertebroplasty using osteoconductive granular material. Spine (Phila Pa 1976).

[33] Heo DH, Kuh SU (2007). Progressive, repeated lumbar compression fracture at the same level after vertebral kyphoplasty with calcium phosphate cement: case report. J Neurosurg Spine.

[34] Perry A, Mahar A, Massie J (2005). Biomechanical evaluation of kyphoplasty with calcium sulfate cement in a cadaveric osteoporotic vertebral compression fracture model. Spine J.

[35] Wang ML, Massie J, Perry A, Garfin SR, Kim CW (2007). A rat osteoporotic spine model for the evaluation of bioresorbable bone cements. Spine J.

[36] Krebs J, Aebli N, Goss BG (2007). Cardiovascular changes after pulmonary embolism from injecting calcium phosphate cement. J Biomed Mater Res B Appl Biomater.

[37] Belkoff SM, Mathis JM, Jasper LE, Deramond H (2001). An ex vivo biomechanical evaluation of a hydroxyapatite cement for use with vertebroplasty. Spine (Phila Pa 1976).

[38] Rao RD, Singrakhia MD (2003). Painful osteoporotic vertebral fracture. Pathogenesis, evaluation, and roles of vertebroplasty and kyphoplasty in its management. J Bone Joint Surg Am.

